This article has been retracted.

# The Pathogenesis and Influencing Factors of Adult Hypertension Based on Structural Equation Scanning

**DOI:** 10.1155/2022/2663604

**Published:** 2022-05-27

**Authors:** Yaqiong Wu, Guangyu Ma, Nana Feng, Zhiqiang Zhang, Sijie Zhang, Xingtao Li

**Affiliations:** ^1^The Department of Cardiology, Fourth Hospital of Hebei Medical University, Shijiazhuang, Hebei 050011, China; ^2^The Department of Haematology, Fourth Hospital of Hebei Medical University, Shijiazhuang, Hebei 050011, China

## Abstract

Explore the pathogenesis and influencing factors of adult hypertension based on structural equation scanning. Using a multistage random sampling method, randomly select 2 community health service centers in each administrative area of a certain city and conduct a sample survey of residents in the community. According to the predetermined sample size *n*, multiply by 1.3 (1.3*n*) to draw a sample. Community doctors and medical students who have been uniformly trained form an investigation team draw up a questionnaire by consulting the literature, seek expert opinions, and then make changes based on the questions in the preinvestigation. Experiment result shows that the average systolic blood pressure of the experimental subjects was 126.13 + 15.36 mmHg and the average diastolic blood pressure was 79.52 + 8.81 mmHg; males are higher than females and increase with age. The prevalence rate of hyperemia is 26.3%, and the prevalence rate of prehypertension among the survey subjects is 55.4%; that of males (62.6%) is higher than that of females (49.2%). The prevalence of isolated systolic hypertension was 7.5%, and that of men (6.9%) was lower than that of women (7.9%). The awareness rate of hypertension was 66.5%, and the treatment rate of hypertension was 62.7%; the control rate of hypertension was 13.2%, and the control rate of hypertension treatment was 25.7%; all the abovementioned rates are higher for women than for men, and they all tend to increase with age which proved that being overweight is a risk factor for hypertension, dyslipidemia, and hypertension. Hypertension, dyslipidemia, and family history of hypertension are risk factors for hypertension. There is a positive correlation between hypertension and dyslipidemia.

## 1. Introduction

Hypertension refers to the increase in systemic arterial blood pressure (systolic blood pressure and/or diastolic blood pressure) (systolic blood pressure ≥ 140 mmHg (1 mmHg = 0.133 kPa), diastolic blood pressure ≥ 90 mmHg) which is the main feature; it may be accompanied by clinical syndromes of organ function or organic damage such as that in the heart, brain, and kidney. Hypertension is currently one of the main diseases threatening human health, it not only caused serious physical, mental, and economic damage to patients but also brings a significant economic burden of disease to all mankind. Hypertension is a disease caused by multiple causes; according to research, hypertension is affected by the interaction of genetic, social, and lifestyle factors, with the improvement of living standards; the choice of diet has increased; obesity among adolescents is also increasing; as a result, hypertensive patients are gradually becoming youthful, which further makes hypertension an important public health problem [1]. In addition, the complications caused by high blood pressure cannot be ignored; in China, hypertension combined with coronary heart disease is more common. As a kind of high blood pressure, it has obvious characteristics of high blood pressure; the quality of life of patients can be improved by improving living habits after the onset of disease. With the development of social economy and the progress of urbanization, with the increase in life expectancy, the problem of population aging has become more and more serious [2]. According to the China Health Service Survey, the prevalence of hypertension in middle-aged and elderly people is gradually increasing and the phenomenon of multiple types of hypertension in the elderly is becoming more and more serious; it has become a major public health problem in China. There are many factors that affect the number of hypertension in the elderly; previous studies only analyzed the direct effects of related influencing factors on the number of hypertension; the interaction between factors and the indirect effects on outcome variables are ignored. Structural equation scanning modeling can incorporate multiple variables into the model at the same time and observe the interaction between various variables and the direct or indirect effects on the outcome variables; it can fully explain the influence of research factors on outcome variables.

With the rapid increase in the prevalence of hypertension, the disability, death, and related diseases caused by it have greatly threatened the health and social and economic development of Chinese residents. What is more worrying is that among hypertensive patients, less than 50% of hypertensive patients know that they are sick; only 25% of those are taking medication and control blood pressure to less than 10% of the normal range. The high prevalence, low awareness, treatment, and control rates of hypertension have become the bottleneck for the prevention and treatment of cardiovascular disease in China [3]. In response to this research question, according to Duarte and others, being overweight or obesity is one of the important factors for elevated blood pressure, regardless of whether children or adults; body weight is highly correlated with blood pressure. Relevant information shows that those who are overweight and have a family history of hypertension may have a dual effect, which will have a synergistic effect [4]. The body mass index of most individuals has a significant correlation with the percentage of body fat; it can better reflect the degree of obesity of the body. Increased body mass index is an independent risk factor for hypertension. Wang et al. believe that dietary factors are the most important environmental factors related to cardiovascular disease [5]. Although the Chinese diet is low in fat compared to the Western diet, low saturated fat and low cholesterol help to keep serum cholesterol and body mass index at a low level, but at the same time, China's low-calcium, low-potassium, and low-animal protein diets also promote the blood pressure effect of sodium. Therefore, the Chinese diet based on plant foods has many factors that promote blood pressure and has a lack of protective factors; this may be the reason why the Chinese population who has been exposed to high sodium for a long time has a greater slope of blood pressure with age than other populations. The influence of dietary factors on blood pressure is the result of the combined effect of many factors [6]. According to Diederichs and Neuhauser, the main risk factors for male hypertension are BMI and salt intake; the main risk factors for women are serum total cholesterol, age, and BMI; the content of total cholesterol in serum is affected by the intake of meat, fish, and green vegetables. Salt intake is positively correlated with high blood pressure in men, but there is no such relationship in women [7].

Based on the current research, this paper investigates the influence of social and economic background on overweight, hypertension, dyslipidemia and hypertension through individual lifestyle behaviors, such as smoking, drinking, exercise and salt intake, through a sample survey of community residents in a city. The main findings are as follows: family history of hypertension, dyslipidemia, hypertension, overweight, and lifestyle behavior (salt intake, active exercise, drinking, and smoking) are risk factors for hypertension.

## 2. Method

### 2.1. Experimental Subjects

The survey object is the permanent population of a certain urban area, aged 18–80 years. Two community health service centers were randomly selected from each district, and samples were drawn according to the predetermined sample content *n*, multiplied by 1.2 (1.2*n*). The respondent was asked to sit and rest for 5 minutes before measuring blood pressure and asked if they smoked or drank within half an hour before the measurement; those who smoked or drank within half an hour were excluded and included in the analysis; all respondents signed an informed consent form.

### 2.2. Principle of the Structural Equation Scanning Model

Structural equation scanning modeling introduces path analysis into hidden variables; at the same time, using the method of factor analysis, the hidden variables and the observed variables are effectively combined and the multivariate statistical analysis method is proposed [8]. It is an analysis method that combines factor *H*_0_ : *F*_*A*_ = *F*_*B*_ analysis and path analysis; compared with traditional analysis methods, it can handle the relationship between multiple dependent variables and independent variables at the same time and clarify the relationship structure between factors [9].

The structural equation scanning model consists of two parts, the measurement model and the structural model.

The measurement model is equivalent to factor analysis, which can explain the subordination between the measured variable and the latent variable of its response, and its equation is expressed as

(1) $$\begin{array}{c} x=A_{x}\xi +\delta ,\\ y=A_{y}\eta +\varepsilon . \end{array}$$

*x*, *y* represent exogenous and endogenous measurement variables, respectively, *ξ*, *η* are exogenous and endogenous latent variables, respectively; *A*_*x*_, *A*_*y*_ are the relationship between exogenous measured variables and latent variables and endogenous measured variables and latent variables; *A*_*x*_ is the factor loading matrix of the exogenous index on the exogenous latent variable, and *A*_*y*_ is the factor loading matrix of the endogenous index on the endogenous latent variable; *δ* and *ε* are the error terms of exogenous and endogenous measurement variables. Exogenous means that the factor only affects other factors; it is not affected by other factors. Endogenous means that the factor is affected by other factors and can affect other factors [10].

The structural model is equivalent to path analysis, explaining the relationship between the latent variables, and its equation is expressed as

(2) $$\begin{array}{c} \eta =B\eta +r\xi +\zeta . \end{array}$$

*η* is the endogenous latent variable, *ξ* is the exogenous latent variable, and *B* is the relationship between the endogenous latent variable; *r* is the influence of exogenous latent variables on endogenous latent variables; *ζ* is the residual term of the structural equation scanning, reflecting the part that *η* cannot be explained in the equation [11].

The fitting of the structural equation scanning model requires 8 matrices; in addition to the 4 matrices *A*_*x*_*A*_*y*_*Br* appearing in the abovementioned two models, the other 4 matrices are *Φ* (covariance matrix of exogenous latent variable *ξ*), Ψ (covariance matrix of error variable *ζ*), Θ_*ε*_ (the covariance matrix of the endogenous observation variable error term *ε*), and Θ_*δ*_ (exogenous indicator variable error term *δ* covariance matrix). Through the transformation of these eight matrices, a new variance covariance matrix *S* about *Y* and *X* can be obtained; compare the original data variance covariance matrix with the newly generated matrix *S*, to judge the fitting effect; the closer the two are, the better the fitting effect [12].

The basic principles of the structural equation scanning model can be summarized as two types of variables (explicit variables and latent variables), two models (measurement model and structural model), and two pathways (path between latent and explicit variables and the path between latent variables). Structural equation scanning models can also fit multiple sets of data at the same time. This function is mainly used to test the applicability of the same model among different sample data [13]. At this time, the first thing to check is whether the shape of the model is consistent between different groups (forms)*H*_0_ : *F*_*A*_ = *F*_*B*_, including the number of index variables and latent variables in the model, the subordination relationship, and the structural relationship between the latent variables, only if this condition is met, in order to continue to check whether the covariance matrices of the model parameters are equal (covariance matrices) *H*_0_ : *Σ*_*A*_ = *Σ*_*B*_. Among the various parameters, we must first test the consistency of the load between the latent variable and the index variable (*A*_*X*_, *A*_*y*_). On this basis, it can be tested in turn according to the essence of the research question:

(3) $$\begin{array}{c} H_{0}:B_{A}=B_{B},\\ r_{A}=r_{B},\\ H_{0}:B_{A}=B_{B},\\ r_{A}=r_{B},\\ \Phi_{A}=\Phi_{B},\\ H_{0}:B_{A}=B_{B},\\ r_{A}=r_{B},\\ \Phi_{A}=\Phi_{B},\\ \Psi_{A}=\Psi_{B}. \end{array}$$

In the abovementioned formula, *Φ* is the variance and covariance of the measurement error and Ψ is the variance and covariance of the regression residual. The abovementioned layers are assumed to be nested relationships, based on *H*_0_ : *F*_*A*_ = *F*_*B*_; when the first hypothesis is rejected, the later hypothesis does not need to be tested [14]. When the previous hypothesis is true, it can be tested by the likelihood ratio, that is, the difference of *X*^2^ between two adjacent hypothetical models (Δ*X*^2^) and the difference of degrees of freedom (Δ*df*) to determine; set whether there is a difference between the new model formed by an equal part of the parameters and the previous model. If the likelihood ratio result is significant, it means that there are differences between the two models with nested relationships and the research hypothesis corresponding to the second model is rejected [15].

The evaluation of the structural equation scanning model is mainly based on the index of goodness of fit that cannot meet the corresponding standard. The test of the goodness of fit of the structural equation scanning model is not as straightforward as other multivariate statistical analysis methods, because there is no indicator that can tell whether the model fits correctly, but researchers can compare the goodness of fit of different models based on these indicators. In other words, although the structural model does not provide the final answer to the model setting but it provides the flexibility to form and test various hypothetical models, make the analysis result more fully explain the relationship contained in the data. The goodness of fit test indicators provided by different statistical analysis software are also different.

## 3. Results and Analysis

### 3.1. Smoking

Among the respondents in this survey, the difference in smoking rates between males and females was statistically significant; the smoking rate of men is much higher than that of women. Among men, the smoking rate is highest in middle-aged age and lowest in old age. Among women, the elderly have the highest smoking rate and the young are the lowest. See Table 1 for details.

### 3.2. Prevalence of Hypertension

Among the respondents in this survey, 33.5% of the respondents had a family history of hypertension, the prevalence rate of hypertension was 11.2%, and the rate of dyslipidemia was 5.5%; those with cerebrovascular disease accounted for 4.3%, and those with cardiovascular disease accounted for 7.3%; the prevalence of various types of hypertension in the survey subjects is shown in Table 2 for details.

### 3.3. Effect Decomposition of Factors Affecting Hypertension in Male Population

The standardized total effect shows that the effects of risk factors for hypertension in descending order are as follows: family history of hypertension, overweight, dyslipidemia, hypertension, salt intake, drinking, and active exercise [16]. The effect of the protective factors of hypertension is as follows: high GDP level, high SES level, and smoking. See Figure 1.

### 3.4. Effect Decomposition of Factors Affecting Hypertension in Female Population

The standardized total effect shows that the effects of the risk factors for hypertension, from large to small, are as follows: family history of hypertension, overweight, dyslipidemia, high blood pressure, salt intake, active exercise, and smoking. The effects of the protective factors of hypertension in descending order are as follows: high GDP level, high SES level, and alcohol consumption [17]. See Table 3 for details.

## 4. Discussion

Based on further understanding of prehypertension that the etiological factor model proposes, the causes of diseases include external causes (such as socioeconomic factors, lifestyle, and living environment) and internal proximate causes (such as the pathophysiological changes of the body) [18]. Although these factors are independent of each other but they interact with each other to form a causal chain, that is, a certain factor can be the cause of the change of other factors or it can be the result of other factors, these causal links form the structure of the cause network [19]. Hypertension is a disease caused by the combined action of many factors, and its influencing factors can be divided into personal characteristics (gender, age), socioeconomic background (living environment, culture, and income level), behavioral factors (smoking, drinking, insufficient exercise, and high-salt diet), and health factors (hyperglycemia, dyslipidemia, and obesity). These factors are connected to each other and have an effect on human health [20]. In the relationship between life behavior style and hypertension involved in this study, the direct effect of salt intake on hypertension is statistically significant; however, the direct effects of active exercise, smoking, and drinking on hypertension were not statistically significant. This situation may be due to the structural equation scanning model analysis; the relationship between a certain factor and the disease includes two parts, a direct effect and an indirect effect; when other mediating factors are included in the model, the direct effects will be weakened or even disappear. In addition to the direct effect of lifestyle on hypertension in this study, it also has an indirect effect on high blood pressure through being overweight, high blood pressure, and dyslipidemia; it may be that these indirect effects through intermediary factors which explain part of the relationship between lifestyle and hypertension. In addition, although community residents' awareness, treatment, and control of hypertension have improved but for blood pressure prevention and control, we still have a lot of work to do and need to further strengthen the health education of hypertension-related knowledge; in the future, further research will be conducted on related factors affecting blood pressure control to help patients control blood pressure levels more effectively [21].

Studies have found that the sleep quality, as a variable factor, has a protective effect on the number of hypertension. Gender, age, and ethnicity have a direct or indirect effect on the number of hypertension; the path coefficients of these factors are small, which still suggests that in the prevention and control of hypertension, corresponding intervention measures should be taken for the relevant behavioral risk factors among elderly people of different ages, ethnicities, and genders. Studies have found that with increasing age, the proportion of the elderly who lack physical activity has increased. At the same time, as the age increases, the socioeconomic status of the elderly declines; it is a risk factor for the increase in the number of hypertension. Therefore, in the prevention and control of hypertension, for the elderly, the government should increase subsidies, improve the economic conditions of the elderly while strengthening social support, pay attention to family care of the elderly, improve the emotional and physical state of the elderly, improve the quality of sleep, and encourage the elderly to exercise properly. For female obesity, the central obesity rate is high, the socioeconomic status is low, and the influence of these pathways has led to an increase in the number of hypertension. Therefore, in rural survey areas, elderly women with low socioeconomic status and obesity or central obesity are the key populations for the prevention and control of hypertension; in the prevention and control of hypertension, this group should be targeted, carry out health education, improve the welfare of the elderly, and prevent the occurrence of hypertension [22].

## 5. Conclusion

The results of a sample survey of residents aged 18–80 years in a certain city's community showed that, in the structural equation scanning by gender, the model has the same appearance between the male and female groups but the path coefficients are not consistent. SES and GDP indirectly affect hypertension through behavior and health status; it also has a direct impact on the distribution of hypertension; it suggests that external socioeconomic background factors also play an important role in the development of the disease. The socioeconomic background affects being overweight, hypertension, dyslipidemia, and hypertension through personal lifestyle behaviors such as smoking, drinking, exercise, and salt intake. The main findings are as follows: family history of hypertension, dyslipidemia, hypertension, overweight, and lifestyle behavior (salt intake, active exercise, drinking, and smoking) are risk factors for hypertension. The hypothesis that external causes (social and economic background) affect the occurrence of diseases through internal proximate causes (behavior, health status) is verified.

## Figures and Tables

**Figure 1:** Decomposition of effects of factors affecting hypertension in males.

**Table 1:** Analysis of smoking status among study subjects of different ages and genders.

Age group	Man		Women	
	Number of people	Smoking rate	Number of people	Number of people
Youth	4975	45.8	5335	2.8
Middle aged	4720	55.2	5324	5.1
Elderly	2120	27.1	2360	13.5

**Table 2:** The prevalence of various types of hypertension in the study subjects.

Hypertension	Number of patients	Prevalence (%)
Hypertension	2585	11.2
Dyslipidemia	1431	5.5
Hypertensive nephropathy	108	0.6
Impaired kidney function	66	0.2
Ischemic stroke	662	2.9
Cerebral hemorrhage	140	0.8
Transient ischemic attack	122	0.6
Myocardial infarction	260	1.2
Angina pectoris	725	3.2
Coronary revascularization	391	1.8
Congestive heart failure	252	1.1
Peripheral vascular disease	40	0.5

**Table 3:** Effect decomposition of factors affecting hypertension in female population.

Variable	Direct effect	Indirect effect	Standard direct effect	Standard indirect effect
CDP	−0.019	−0.002	−0.026	−0.005
SES	−0.012	—	−0.030	−0.002
Smoking	0.022	−0.006	0.013	−0.004
Drinking	−0.006	0.004	−0.002	0.005
Active exercise	0.004	0.005	0.005	0.006
Salt intake	0.018	0.002	0.021	0.002
Overweight	0.082	0.015	0.142	0.020
Dyslipidemia	0.168	—	0.122	—
Hypertension	0.148	—	0.078	—

## Data Availability

The data used to support the findings of this study are available from the corresponding author upon request.
